# Dose–Volume and Radiobiological Model-Based Comparative Evaluation of the Gastrointestinal Toxicity Risk of Photon and Proton Irradiation Plans in Localized Pancreatic Cancer Without Distant Metastasis

**DOI:** 10.3389/fonc.2020.517061

**Published:** 2020-10-23

**Authors:** Vijay P. Raturi, Taku Tochinai, Hidehiro Hojo, Toshiya Rachi, Kenji Hotta, Naoki Nakamura, Sadamoto Zenda, Atsushi Motegi, Takaki Ariji, Yasuhiro Hirano, Hiromi Baba, Hajime Ohyoshi, Masaki Nakamura, Masayuki Okumura, Yanping Bei, Tetsuo Akimoto

**Affiliations:** ^1^Division of Radiation Oncology and Particle Therapy, National Cancer Center Hospital, Chiba, Japan; ^2^Course of Advanced Clinical Research of Cancer, Graduate School of Medicine, Juntendo University, Tokyo, Japan

**Keywords:** pancreatic cancer, normal tissue complication probability (NTCP), intensity modulated radiation therapy (IMRT), volumetric modulated arc therapy (VMAT), proton beam therapy (PBT), dosimetry

## Abstract

**Background:** Radiobiological model-based studies of photon-modulated radiotherapy for pancreatic cancer have reported reduced gastrointestinal (GI) toxicity, although the risk is still high. The purpose of this study was to investigate the potential of 3D-passive scattering proton beam therapy (3D-PSPBT) in limiting GI organ at risk (OAR) toxicity in localized pancreatic cancer based on dosimetric data and the normal tissue complication probability (NTCP) model.

**Methods:** The data of 24 pancreatic cancer patients were retrospectively analyzed, and these patients were planned with intensity-modulated radiotherapy (IMRT), volume-modulated arc therapy (VMAT), and 3D-PSPBT. The tumor was targeted without elective nodal coverage. All generated plans consisted of a 50.4-GyE (Gray equivalent) dose in 28 fractions with equivalent OAR constraints, and they were normalized to cover 50% of the planning treatment volume (PTV) with 100% of the prescription dose. Physical dose distributions were evaluated. GI-OAR toxicity risk for different endpoints was estimated by using published NTCP Lyman–Kutcher–Burman (LKB) models. Analysis of variance (ANOVA) was performed to compare the dosimetric data, and ΔNTCP_IMRT−PSPBT_ and ΔNTCP_VMAT−PSPBT_ were also computed.

**Results:** Similar homogeneity and conformity for the clinical target volume (CTV) and PTV were exhibited by all three planning techniques (*P* > 0.05). 3D-PSPBT resulted in a significant dose reduction for GI-OARs in both the low-intermediate dose range (below 30 GyE) and the highest dose region (*D*_max_ and *V*_50 GyE_) in comparison with IMRT and VMAT (*P* < 0.05). Based on the NTCP evaluation, the NTCP reduction for GI-OARs by 3D-PSPBT was minimal in comparison with IMRT and VMAT.

**Conclusion:** 3D-PSPBT results in minimal NTCP reduction and has less potential to substantially reduce the toxicity risk of upper GI bleeding, ulceration, obstruction, and perforation endpoints compared to IMRT and VMAT. 3D-PSPBT may have the potential to reduce acute dose-limiting toxicity in the form of nausea, vomiting, and diarrhea by reducing the GI-OAR treated volume in the low-to-intermediate dose range. However, this result needs to be further evaluated in future clinical studies.

## Introduction

Pancreatic cancer is a lethal malignancy with a high mortality rate. In Japan, pancreatic cancer is the fourth primary cause of cancer-related deaths, and the age-standardized (world) mortality rate was 7.8 age-standardized rate (ASR) per 100,000 in 2018 (1, 2). Pancreatic ductal adenocarcinoma (PDAC) is the most common type of pancreatic cancer (3). Localized PDAC has been classified into resectable, borderline resectable (BR), and locally advanced/unresectable pancreatic cancer (LAPC) (4).

In the long term, surgical resection can offer a possibility of better survival; however, <20% of patients are initially diagnosed with resectable disease. The 5-year overall survival (OS) rate for the entire patient population is <5%. Chemoradiotherapy (CRT) has played a key role in the therapeutic management of LAPC for the last two decades (5, 6). As reported by many studies, the surgical resection rates and the histological treatment response after neoadjuvant regimens that have incorporated radiotherapy (RT) seem to be higher in BR patients than after neoadjuvant chemotherapy alone, with no differences in the survival rates (7–9).

Technological advancements in RT delivery over the past decade have resulted in better tumor targeting and conformity. Dosimetric studies have reported improved target coverage and better sparing of organs at risk (OARs) by using newer radiation treatment modalities such as intensity-modulated radiotherapy (IMRT) and volumetric-modulated arc therapy (VMAT) (10, 11). Charged particles, such as protons, deposit low-dose energy initially, which is followed by a surge in energy deposition lastly of their course, known as Bragg peak (12). In homogeneous tissues, protons of a particular energy level have a determined range, and there is no exit dose right after the Bragg peak. During treatment, protons with different energies are totaled together to produce a spread-out Bragg peak because the peak occurs over a small distance (13) Thus, 3D-passive scattering proton beam therapy (3D-PSPBT) may provide an advantage over IMRT and VMAT in sparing gastrointestinal (GI)-OARs during RT treatment of pancreatic cancer.

It is often difficult to rank plans based only on dosimetric comparisons using few dose–volume histogram (DVH) data points. Sometimes, even though a statistically significant dosimetric reduction of OAR is reported, it may not translate into considerable differences clinically. Nevertheless, by analyzing the DVH data, the normal tissue complication probability (NTCP) radiobiological model evaluates the treatment plans by using parameters derived from toxicity rates observed in published trials. Careful comparisons between predicted complications and the observed toxicity rates are necessary to validate each set of NTCP parameters found in the literature. Each parameter set is specific for definite endpoints and is patient cohort-and treatment technique-dependent (14). Quantitative analysis using the NTCP model with different toxicity endpoints can provide the link between the physical dose distribution and the expected clinical toxicity. It is more robust than a DVH parameter for investigating GI-OAR-related toxicity, and NTCP evaluation is consistent with and supportive of the so-called radiobiological model-based approach to radiotherapy patient selection (15).

In this study, we performed a dosimetric and radiobiological model-based comparison between IMRT, VMAT, and 3D-PSPBT in patients with localized pancreatic cancer without distant metastasis to assess the potential of 3D-PSPBT as a means of reducing GI-OAR-related toxicity.

## Materials and Methods

With the approval of the Institutional Research Ethics Committee (reference number 2017-440), we analyzed the data of 24 consecutive patients with BR and LAPC without distant metastasis treated at a single institution between 2014 and 2018. Computed tomography (CT) simulation scans were obtained for these 24 patients.

### Volume Definition

The planned treatment area was the primary tumor and positive lymph nodes, and no elective nodal region was included for planning in this study. CT slice thickness was 1–3 mm. The gross tumor volume (GTV) consisted of a visible tumor contoured on each axial CT slice. The clinical target volume (CTV) consisted of the GTV plus a 0.5-cm uniform margin. A CTV-to-PTV expansion of about 1 cm laterally and about 1 cm superoinferiorly was provided for treatment planning purposes. A single observer contoured all plans.

The OARs were contoured for each patient and included the whole stomach, duodenum, small bowel, both kidneys, liver, and the spinal cord. The duodenum was contoured from the pylorus to the ligament of Treitz. The small bowel contour was defined as bowel loops 2 cm superior-inferiorly to the PTV (16). Kidney contours included both the kidney parenchyma. The whole liver was contoured, including the hepatic blood vessels and the intraductal biliary system.

### Treatment Planning

The steps performed in this study are shown in Figure 1. Three plans were generated for each patient (IMRT plan, VMAT plan, and 3D-PSPBT plan), and all 72 plans were analyzed. All our plan calculations were based on the expiratory phase CT dataset. The IMRT and VMAT plans were generated by using the Raystation v6.2 (RaySearch Laboratories, Stockholm, Sweden) treatment planning system (TPS) with a collapsed-cone convolution superposition (CCC v3.4)-based algorithm calculation by setting a dose grid of 0.2 × 0.2 × 0.2 cm^3^. The dynamic multi-leaf collimator (MLC) delivery mode was used for the IMRT and VMAT plans. Non-coplanar 4π IMRT plans were made using six (10 MV beam energy) beams: four coplanar (gantry angles at 30, 90, 175, and 310 with couch at 0) and two non-coplanar beams (gantry at 20 and 330 with couch at 90). For the VMAT plans, two 10-MV full coplanar arcs (181–179) were planned, as shown in Figure 2. The IMRT and VMAT beam modeling was performed for the TrueBeam RT system (Varian Medical System, Inc., Palo Alto, CA). The IMRT and VMAT plans were optimized by using objective functions, dose constraints, and ring regions of interest (ROIs) by the trial-and-error method. 3D-PSPBT plans were generated by using the clinical TPS PTPLAN, version 2.0.1 software (Sumitomo Heavy Industry, Tokyo, Japan) with pencil beam algorithm (PBA) calculation. The TPS PTPLAN does not support robust treatment plan optimization and robust dose analysis. Beam modeling was performed for the proton therapy system (Sumitomo Heavy Industry, Tokyo, Japan). For the proton plans, the distal margin (DM) was set at 0 mm, the proximal margin (PM) at 0 mm, and the compensator smear (CS) at 4.5 mm. Although the DM and PM were set to 0 mm, they were included in the margin because the calculation was performed targeting the PTV. The prescription dose was a uniform 50.4 GyE (Gray equivalent) in 28 fractions. The IMRT, VMAT, and 3D-PSPBT plans were normalized to cover 50% of the PTV with 100% of the prescribed dose. The optimal plans were approved when at least ≥95% of the CTV received ≥95% of the dose, at least ≥95% of the PTV received ≥90% of the dose, and 0% volume of the PTV received <107% of the prescription dose without exceeding the dose constraints of the OARs. The IMRT, VMAT, and 3D-PSPBT plan evaluations were made for nominal dose distributions. All plans were optimized in consensus: the chief photon physicist generated all IMRT and VMAT plans, and another chief proton physicist generated all of the 3D-PSPBT plans. Two physicians checked all of the plans.

**Figure 1:** Steps in dosimetric and normal tissue complication probability (NTCP) evaluation of the intensity-modulated radiotherapy (IMRT), volume-modulated arc therapy (VMAT), and 3D-passive scattering proton beam therapy (3D-PSPBT) plans.

**Figure 2:** Beam directions of all three plans for one representative patient. Axial, sagittal, and coronal CT slices showing the dose distributions of the **(A)** 3D-passive scattering proton beam therapy (3D-PSPBT) plan, **(B)** intensity-modulated radiotherapy (IMRT) plan, and **(C)** volume-modulated arc therapy (VMAT) plan for one representative patient.

The 3D-PSPBT plans were made by using two or three ports (6, 17–19). During 3D-PSPBT planning, the beam directions were chosen so that they would avoid entering the sites where the proton beam would travel through a substantial amount of bowel before reaching the target, e.g., by selecting the posterior, right posterior oblique, and right lateral typical beam angles for pancreatic cancer. The beam range was modified, or different beam angles were used to recompute the proton plan whenever the validation plans demonstrated inadmissible DVH values at the typical beam angles. Based on the study by Uzawa et al. the proton beam output was modulated with a relative biological effectiveness (RBE) of 1.1 (20). As all tissues were presumed to have nearly the same RBE, the doses stated in Gray equivalent are directly in comparison with the photon doses.

The OAR dose constraints for all of the plans were based on the guideline proposed in the study by Ben-Josef et al. (21) and Nevinny-Stickel et al. (22). The maximum dose to the stomach and small intestine was limited to ≤54 GyE. For the stomach, the dose constraints were *V*_50 GyE_ ≤2% and *V*_45 GyE_ ≤25%, respectively. The maximum dose to the duodenum was limited to ≤55 GyE. For the duodenum, the constraint was *V*_45 GyE_ ≤33%. For the small bowel, the dose constraints were *V*_50 GyE_ ≤2% and *V*_45 GyE_ ≤25%, respectively. For both kidneys, the dose constraints were *V*_18 GyE_ ≤50% and *V*_23 GyE_ ≤30%, respectively. The mean liver goal was ≤30 GyE. The maximum dose to the spinal cord was limited to ≤45 GyE.

### Plan Comparisons

The three different plans were compared with respect to target conformity and homogeneity. DVH values for target coverage and OARs were recorded for reporting purposes. Conformity around the CTV and PTV was assessed by using the conformation number (CN) formulas [(CTV95^2^)/(CTV^*^V95)] and [(PTV95^2^)/(PTV^*^V95)], respectively, where CTV95 and PTV95 are the target volumes covered by 95% of the reference isodose, CTV and PTV are target volumes, and V95 is the 95% isodose volume. The CN takes into account the irradiation of the target volume and healthy tissues. A plan is considered increasingly conformal as the CN value approaches 1, and it corresponds to a target volume precisely covered by the 95% isodose line. A CN value of 0 indicates a total absence of conformation or a huge volume of irradiation compared to the target volume (23). Dose homogeneity means the consistency of dose distribution within the target volume. The homogeneity index (HI) was calculated using the RTOG formula [(D2–D98%)/D50%] (24). D2%, D98%, and D50% are the doses received by 2, 98, and 50%, respectively, of the target volume. A HI value of zero indicates that the absorbed dose distribution is almost homogeneous.

### Normal Tissue Complication Probability Evaluation

The Digital Imaging and Communications in Medicine (DICOM) standard RT doses from the IMRT, VMAT, and 3D-PSPBT plans were transferred to MIM (v6.86, MIM Software Inc., Cleveland, OH). The cumulative physical dose was converted into the equivalent dose of 2 Gy (EQD2) per fraction by using a linear-quadratic (LQ) equation with α/β = 4 for the stomach, duodenum, small bowel, and stoduo) before NTCP calculation.

The GI toxicity risk endpoints were computed using the Lyman–Kutcher–Burman (LKB) NTCP model with parameter values taken from the studies by Pan et al., Burman et al., and Holyoake et al., as shown in Table 1 (25–27). NTCP_LKB_ is described using the following equations:

(1) $$\begin{array}{l} \text{NTCP}=\frac{1}{\sqrt{2\pi }}\int_{-\infty }^{t}e^{-\frac{t^{2}}{2}}\;dx \end{array}$$

(2) $$t=\frac{(D_{eff}\;-\;{\text{TD}}_{50)}}{m{\text{TD}}_{50}}$$

(3) $$\begin{array}{l} D_{\text{eff}}={\left(\underset{i}{\sum }v_{i}{D_{i}}^{\frac{1}{n}}\right)}^{n} \end{array}$$

where *D*_eff_ is identical to an equivalent uniform dose (EUD) and TD_50_ is the tolerance dose yielding a 50% complication rate in the normal organ. The parameter *m* represents the slope of the sigmoid dose–response curve and the fractional volume of the organ is represented by *v*_*i*_ receiving a dose *D*_*i*_. The parameter *n* represents the magnitude of the volume effect and (*D*_*i*_, *v*_*i*_) are the bins of differential DVH. The computed NTCP values were used in a relative sense for comparisons between IMRT, VMAT, and 3D-PSPBT. All NTCPs were computed from EQD2 DVH's ASCII files by using RADBIOMOD software (28). Reductions in NTCP provided by 3D-PSPBT in comparison with IMRT (ΔNTCP_IMRT−PSPBT_) and VMAT (ΔNTCP_IMRT−PSPBT_) were also computed.

**Table 1:** Normal tissue complication probability (NTCP) Lyman–Kutcher–Burman (LKB) model parameters used in the biological evaluation of the intensity-modulated radiotherapy (IMRT), volume-modulated arc therapy (VMAT), and 3D-passive scattering proton beam therapy (3D-PSPBT) plans.

**Gastrointestinal OAR (reference)**	**TD_**50**_ (Gy) (range)**	***m* (range)**	***n* (range)**	**Endpoint**
Stomach wall [Pan et al. (25)]	62 (53–71)	0.30 (0.23–0.39)	0.07 (0.03–0.16)	Gastric bleed
Stomach wall [Burman et al. (26)]	65	0.14	0.15	Ulceration/perforation
Duodenum [Pan et al. (25)]	180 (100 to >200)	0.39 (0.36–0.61)	0.12 (0.09–0.30)	Gastric bleed
Duodenum [Holyoake et al. (27)]	299.1	0.51	0.193	Grade ≥3 GI toxicity
Small bowel loops [Burman et al. (26)]	55	0.16	0.15	Obstruction/perforation
Stoduo [Pan et al. (25)]	52.5 (42–64)	0.35 (0.28–0.47)	0.21 (0.11–0.50)	Gastric bleed

*TD_50_, dose at which there is 50% chance of complication; m, slope of the dose–response curve; n, dose–volume relationship*.

### Statistical Analysis

R commander EZR version 2.6-2 software (R version 3.6.3) was used to make all statistical calculations (29). Repeated measures analysis of variance (ANOVA) was used to compare the three techniques. Differences between the pairs of techniques were tested by using the Bonferroni *post-hoc* test. *P* < 0.05 were considered to be statistically significant.

## Results

Patient characteristics are shown in Table 2. The CTV and PTV (mean ± SD) were 79.90 ± 46.85 and 198.06 ± 74.04 cc, respectively. The percentages of PTV overlap (mean ± SD) with the stomach, duodenum, and small bowel were 7.15 ± 5.77, 5.52 ± 5.24, and 2.76 ± 2.01%, respectively.

**Table 2:** Patient characteristics.

**Cases**	**Age (years)**	**Sex**	**TNM stage^**a**^**	**Localized PDAC (location)**	**CTV volume (cc)**	**PTV volume (cc)**	**% PTV overlap with GI-OARs**		
							**Stomach**	**Duodenum**	**Small bowel**
1	65	M	T4N1	LA (body)	198.6	356.5	+ (2.35)	+ (1.07)	+ (2.27)
2	47	M	T3N0	BR (head)	70.7	215.0	+ (0.15)	+ (11.02)	+ (4.45)
3	49	F	T4N0	BR (body)	91.9	291.9	+ (8.80)	–	+ (4.27)
4	75	F	T4N0	LA (head)	70.8	222.9	+ (5.87)	+ (3.18)	+ (2.08)
5	83	M	T3N0	LA (head)	39.8	144.8	+ (1.70)	+ (5.93)	–
6	56	M	T2N1	LA (head)	107.2	298.5	+ (3.69)	+ (5.54)	+ (1.38)
7	77	M	T4N0	LA (body)	57.1	129.7	+ (7.53)	+ (2.36)	+ (0.98)
8	70	F	T4N0	BR (head)	53.5	190.8	+ (5.12)	+ (1.60)	+ (0.67)
9	76	M	T2N1	BR (head)	39.6	167.5	+ (8.38)	+ (7.76)	+ (0.10)
10	52	F	T4N0	LA (head)	70.5	145.4	+ (8.48)	+ (2.02)	+ (2.13)
11	84	M	T4N1	LA (body)	84.2	154.8	+ (10.89)	–	–
12	75	F	T3N0	BR (head)	23.2	95.2	–	+ (21.11)	+ (0.44)
13	56	M	T3N0	LA (head)	116.8	191.3	+ (2.89)	+ (6.45)	+ (2.94)
14	62	M	T3N0	BR (head)	56.9	176.7	+ (5.03)	+ (9.71)	+ (2.93)
15	78	F	T4N0	LA (head)	120.7	179.1	–	+ (11.56)	+ (0.46)
16	71	F	T4N0	LA (body)	32.2	127.0	+ (19.55)	+ (1.12)	+ (5.19)
17	69	M	T4N1	LA (body)	173.8	312.2	–	+ (1.82)	+ (2.41)
18	78	F	T4N0	BR (body)	63.1	265.2	+ (23.83)	+ (0.91)	+ (5.02)
19	77	F	T3N0	BR (body)	33.6	119.5	+ (3.49)	+ (0.38)	+ (6.18)
20	62	M	T4N0	BR (head)	53.2	169.8	+ (2.14)	+ (12.24)	+ (4.25)
21	56	M	T3N0	BR (body)	24.9	82.3	–	–	+ (1.24)
22	69	F	T3N0	BR (body)	157.8	314.3	+ (8.39)	+ (1.10)	+ (6.82)
23	75	F	T4N0	BR (head)	105.2	194.1	+ (7.72)	+ (6.30)	+ (4.29)
24	75	F	T2N1	BR (head)	72.5	209.1	+ (7.14)	+ (2.86)	+ (0.33)

*M, male; F, female; PDAC, pancreatic ductal adenocarcinoma; BR, borderline resectable; LA, locally advanced; CTV, clinical target volume; PTV, planning treatment volume; GI-OAR, gastrointestinal organ at risk; +, overlap seen between PTV and GI-OAR; –, no overlap between PTV and GI-OAR*.

a *Staging was according to the American Joint Committee on Cancer guideline (7th edition manual, 2010)*.

### CTV and PTV Coverage

The average cumulative DVHs for the CTV and PTV in each IMRT, VMAT, and 3D-PSPBT cohort are shown in Figures 3A,B. In accordance with the study protocol for CTV (*V*_95%_ ≥ 95%), all three treatment techniques covered the CTV in all patients appropriately. The PTV coverage goal (*V*_90%_ ≥ 95%) was not met in two patients due to completely abiding by the GI-OAR dose constraints.

**Figure 3:** Average cumulative dose–volume histogram (DVH) of each plan in each cohort for tumor volumes [CTV **(A)** and PTV **(B)**] and gastrointestinal organs at risk (GI-OARs) [stomach **(C)**, duodenum **(D)**, small bowel **(E)**, and stoduo **(F)**]. *Yellow*, 3D-passive scattering proton beam therapy (3D-PSPBT); *magenta*, intensity-modulated radiotherapy (IMRT); *purple*, volume-modulated arc therapy (VMAT).

### Conformity and Homogeneity for CTV and PTV

The results of calculations of the CN values for CTV and PTV and the HIs are shown in Table 3. Similar CTV and PTV homogeneity and conformity were obtained with all three plans (*P* > 0.05).

**Table 3:** Comparison of the target homogeneity and conformity data and the organ at risk (OAR) dosimetric data obtained with the intensity-modulated radiotherapy (IMRT), volume-modulated arc therapy (VMAT), and 3D-passive scattering proton beam therapy (3D-PSPBT) plans.

**Dosimetric parameters**	**Treatment modality**			**Pairwise comparisons**		
	**IMRT (mean ± SD)**	**VMAT (mean ± SD)**	**3D-PSPBT (mean ± SD)**	**IMRT *vs*. VMAT**	**3D-PSPBT *vs*. IMRT**	**3D-PSPBT *vs*. VMAT**
**Target HI and CN**						
CTV HI	0.04 ± 0.02	0.04 ± 0.02	0.04 ± 0.02	0.09	1.0	0.11
CTV CN	0.35 ± 0.11	0.36 ± 0.11	0.34 ± 0.11	0.02^*^	0.63	0.07
PTV HI	0.10 ± 0.04	0.10 ± 0.04	0.12 ± 0.09	1.0	1.0	1.0
PTV CN	0.82 ± 0.04	0.81 ± 0.03	0.81 ± 0.05	0.32	0.25	1.0
**Stomach**						
*D*_max_ (GyE)	52.4 ± 0.83	52.1 ± 0.77	50.3 ± 1.65	0.01^*^	<0.001^*^	<0.001^*^
V_50 GyE_	1.3 ± 0.8%	1.4 ± 0.7%	0.8 ± 0.7%	0.33	0.006^*^	<0.001^*^
V_45 GyE_	8.1 ± 6.4%	7.7 ± 5.7%	7.3 ± 49%	0.64	0.84	1.0
V_40 GyE_	11.3 ± 8.1%	11.2 ± 7.8%	10.6 ± 7.1%	1.0	1.0	1.0
V_35 GyE_	14.9 ± 9.9%	15.1 ± 10.1%	13.6 ± 9.2%	1.0	0.65	0.50
V_30 GyE_	19.1 ± 12.4%	20.2 ± 13.2%	16.4 ± 10.8%	0.05	0.03^*^	0.008^*^
V_25 GyE_	24.3 ± 15.0%	26.9 ± 16.9%	21.7 ± 15.5%	0.002^*^	0.92	0.15
V_20 GyE_	32.9 ± 18.8%	36.1 ± 0.20%	23.0 ± 14.2%	0.13	<0.001^*^	<0.001^*^
V_15 GyE_	40.5 ± 20.9%	46.1 ± 23.7%	29.1 ± 18.3%	0.03^*^	<0.001^*^	<0.001^*^
V_10 GyE_	47.8 ± 21.5%	52.0 ± 24.4%	38.3 ± 22.0%	0.02^*^	0.007^*^	0.001^*^
V_5 GyE_	56.1 ± 21.9%	59.4 ± 23.3%	44.6 ± 24.2%	0.07	0.004^*^	<0.001^*^
**Duodenum**						
*D*_max_ (GyE)	51.0 ± 8.1	51.1 ± 7.2	48.7 ± 10.4	1.0	0.004^*^	0.008^*^
*V*_50 GyE_	9.9 ± 7.4%	9.7 ± 7.4%	5.7 ± 6.6%	1.0	<0.001^*^	<0.001^*^
*V*_45 GyE_	19.0 ± 12.8%	19.9 ± 12.8%	19.8 ± 12.9%	0.04^*^	0.64	1.0
*V*_40 GyE_	26.4 ± 19.3%	28.5 ± 20.2%	26.1 ± 16.5%	0.008^*^	1.0	0.41
*V*_35 GyE_	32.1 ± 22.6%	35.5 ± 24.5%	31.6 ± 19.9%	0.004^*^	1.0	0.04^*^
*V*_30 GyE_	38.2 ± 25.2%	43.2 ± 26.8%	36.7 ± 23.2%	<0.001^*^	0.65	<0.001^*^
*V*_25 GyE_	45.1 ± 28.0%	53.9 ± 26.1%	41.9 ± 25.5%	<0.001^*^	0.10	<0.001^*^
*V*_20 GyE_	54.1 ± 28.1%	64.0 ± 24.8%	46.8 ± 27.0%	0.01^*^	<0.001^*^	<0.001^*^
*V*_15 GyE_	61.9 ± 28.3%	71.0 ± 21.5%	52.7 ± 28.4%	0.03^*^	0.04^*^	0.003^*^
*V*_10 GyE_	73.7 ± 22.1%	78.1 ± 17.2%	59.8 ± 27.4%	0.23	0.005^*^	0.002^*^
*V*_5 GyE_	84.3 ± 16.8%	82.8 ± 16.1%	64.2 ± 29.1%	0.84	0.001^*^	0.001^*^
**Small bowel**						
*D*_max_ (GyE)	51.7 ± 3.4	51.6 ± 2.9	49.5 ± 3.1	1.0	<0.001^*^	<0.001^*^
*V*_50 GyE_	1.1 ± 0.7%	1.1 ± 0.7%	0.6 ± 0.7%	1.0	0.03^*^	0.01^*^
*V*_45 GyE_	3.1 ± 3.0%	3.3 ± 3.2%	2.9 ± 2.3%	0.14	1.0	1.0
*V*_40 GyE_	4.3 ± 3.8%	4.7 ± 4.2%	4.3 ± 3.2%	0.22	1.0	1.0
*V*_35 GyE_	5.7 ± 4.8%	6.5 ± 5.3%	5.5 ± 2.3%	0.04^*^	0.97	0.99
*V*_30 GyE_	7.5 ± 6.0%	9.1 ± 7.0%	7.6 ± 5.3%	0.005^*^	1.0	0.11
*V*_25 GyE_	12.1 ± 8.0%	13.1 ± 9.2%	9.6 ± 6.6%	0.39	0.01^*^	0.008^*^
*V*_20 GyE_	23.8 ± 11.9%	20.4 ± 11.9%	12.2 ± 7.6%	0.07	<0.001^*^	<0.001^*^
*V*_15 GyE_	30.6 ± 14.3%	31.4 ± 13.7%	15.6 ± 12.2%	1.0	<0.001^*^	<0.001^*^
*V*_10 GyE_	36.3 ± 14.7%	39.5 ± 14.7%	25.8 ± 13.9%	0.13	0.004^*^	<0.001^*^
*V*_5 GyE_	45.2 ± 14.5%	47.3 ± 15.0%	30.0 ± 16.0%	0.16	<0.001^*^	<0.001^*^
**Stoduo**						
*V*_50 GyE_ (cc)	8.59 ± 4.23	8.25 ± 4.28	5.59 ± 4.61	1.0	<0.001^*^	<0.001^*^
**Kidneys**						
*D*_mean_ (GyE)	5.19 ± 2.05	7.10 ± 3.15	4.4 ± 3.81	0.02^*^	0.93	0.02^*^
**Liver**						
*D*_mean_ (GyE)	2.2 ± 2.2	3.75 ± 3.6	3.1 ± 2.9	<0.001^*^	0.13	0.76
**Spinal cord**						
*D*_max_ (GyE)	20.6 ± 3.6	19.3 ± 2.7	14.9 ± 11.4	<0.002^*^	0.03^*^	0.04^*^

*IMRT, intensity-modulated radiotherapy; VMAT, volumetric-modulated arc radiotherapy; 3D-PSPBT, 3D-passive scattering proton beam therapy; CN, conformation number; HI, homogeneity index; GyE, Gray equivalent; V_(X)%_, percentage volume of OAR at or above “X” GyE; D_max_, maximum dose; D_mean_, mean dose; SD, standard deviation*.

* *Significant (P < 0.05)*.

### Doses to the GI Tract and Other Organs at Risk

All dose–volume parameters (mean ± SD) for OARs (stomach, small bowel, duodenum, stoduo, kidneys, liver, and the spinal cord) are shown in Table 3.

3D-PSPBT decreased the stomach, duodenum, and small bowel doses in low-intermediate regions (*P* < 0.05) and showed a clear dosimetric benefit below 30 GyE compared to IMRT and VMAT. However, no significant difference was seen between 3D-PSPBT, IMRT, and VMAT in the dose range above 30 GyE and below 50 GyE. Figures 3C–E depict the average comparative dose–volume relationship between the 3D-PSPBT, IMRT, and VMAT cohorts in more detail. In all cases, 3D-PSPBT also demonstrated a relative superiority in the highest dose region (*V*_50 GyE_) and *D*_max_ for GI-OARs compared to IMRT and VMAT (*P* < 0.05). Using 3D-PSPBT, the *V*_50 GyE_ for stoduo was significantly reduced by ≈35 and ≈32% (5.59 vs. 8.59 cc, *P* < 0.001, and 5.59 *vs*. 8.25 cc, *P* = 0.001) compared to IMRT and VMAT.

Doses to the other OARs, i.e., the kidneys, liver, and spinal cord, were within the dose constraint and did not impose limitations on treatment planning. The *D*_mean_ to the kidneys was reduced by ≈15 and ≈32%, respectively, in the 3D-PSPBT plan in comparison with the IMRT and VMAT plans (4.4 *vs*. 5.19 GyE, *P* = 0.93, and 4.4 vs. 7.10 GyE, *P* = 0.02, respectively). The *D*_mean_ to the liver with IMRT was significantly lower, ≈41% lower, in comparison with VMAT (2.20 *vs*. 3.75 GyE, *P* < 0.001). 3D-PSPBT reduced the spinal cord *D*_max_ significantly in comparison with IMRT (14.9 vs. 20.6 GyE, *P* = 0.03) and VMAT (14.9 vs. 19.3 GyE, *P* = 0.04).

### NTCP Analysis of GI and Other OARs

The NTCP values computed by RADBIOMOD for the liver, kidneys, and the spinal cord of each patient and each of the three plans, IMRT, VMAT, and 3D-PSPBT, were 0%. The NTCP values calculated for the stomach, duodenum, small bowel, and stoduo for the IMRT, VMAT, and 3D-PSPBT plans are shown in Table 4 and Figures 4A–D. The dose reduction of the GI-OARs in the high-dose region of *V*_50 GyE_ and *D*_max_ obtained using 3D-PSPBT did not result in a substantial NTCP reduction in comparison with IMRT and VMAT (Figures 5A–D). The NTCP reduction of 3D-PSPBT (ΔNTCP_IMRT−PSPBT_ and ΔNTCP_VMAT−PSPBT_) was minimal for the upper GI bleeding, ulceration, obstruction, and perforation toxicity endpoints (Table 4). The NTCP values for the gastric ulceration/perforation and small bowel obstruction/perforation endpoints were lower, and similar values were predicted for all techniques (Table 4 and Figures 4A,C).

**Table 4:** Normal tissue complication probability (NTCP) and NTCP reduction (ΔNTCP) of gastrointestinal organ at risk (GI-OAR) radiation-related toxicity compared between the intensity-modulated radiotherapy (IMRT), volume-modulated arc therapy (VMAT), and 3D-passive scattering proton beam therapy (3D-PSPBT) plans.

**Gastrointestinal OAR**	**NTCP (%)**			**ΔNTCP_**IMRT-PSPBT**_ (mean ± SD)**	**ΔNTCP_**VMAT-PSPBT**_ (mean ± SD)**
	**IMRT (mean ± SD)**	**VMAT (mean ± S.D)**	**PSPBT (mean ± S.D)**		
**Stomach wall**					
Ulceration/perforation [Burman et al. (26)]	0.01 ± 0.01%	0.01 ± 0.01%	0.01 ± 0.01%	0.0 ± 0.0%	0.0 ± 0.0%
Gastric bleed [Pan et al. (25)]	8.33 ± 2.79%	8.49 ± 2.59%	8.17 ± 2.87%	0.15 ± 1.0%	0.31 ± 0.98%
**Duodenum**					
Gastric bleed [Pan et al. (25)]	1.93 ± 0.41%	1.95 ± 0.39%	1.88 ± 0.42%	0.0 ± 0.0%	0.0 ± 0.0%
Grade ≥3 GI toxicity [Holyoake et al. (27)]	3.85 ± 0.40%	3.89 ± 0.36%	3.81 ± 0.41%	0.0 ± 0.0%	0.0 ± 0.0%
**Small bowel loops**					
Obstruction/perforation [Burman et al. (26)]	0.11 ± 0.20%	0.08 ± 0.09%	0.05 ± 0.05%	0.0 ± 0.0%	0.0 ± 0.0%
**Stoduo**					
Gastric bleed [Pan et al. (25)]	7.70 ± 2.32%	7.89 ± 2.26%	7.35 ± 2.01%	0.30 ± 0.96%	0.18 ± 0.34%

*ΔNTCP_IMRT−PSPBT_, 3D-PSPBT NTCP reduction in comparison with IMRT; ΔNTCP_VMAT−PSPBT_, 3D-PSPBT NTCP reduction in comparison with VMAT*.

**Figure 4:** Normal tissue complication probability (NTCP, in percent) of gastrointestinal organs at risk (OARs) [stomach **(A)**, duodenum **(B)**, small bowel **(C)**, and stoduo **(D)**] for intensity-modulated radiotherapy (IMRT), volume-modulated arc therapy (VMAT), and 3D-passive scattering proton beam therapy (3D-PSPBT) calculated using Lyman–Kutcher–Burman (LKB) model parameters from Pan et al., Burman et al., and Holyoake et al. (graph: NTCP% is plotted along the *Y*-axis).

**Figure 5:** Normal tissue complication probability (NTCP) reduction (ΔNTCP_Photon−Proton_) of gastrointestinal oragsn at risk (OARs) [stomach **(A)**, duodenum **(B)**, small bowel **(C)**, and stoduo **(D)**] for proton therapy (3D-PSPBT) calculated using Lyman–Kutcher–Burman (LKB) model parameters from Pan et al., Burman et al., and Holyoake et al. (graph: on the *X*-axis are the patient numbers from 1 to 24; on the *Y*-axis are the ΔNTCP_Photon−Proton_ values).

## Discussion

In our study, based on the NTCP calculation and dosimetric assessment, 3D-PSPBT does not result in a decrease in the radiation-related toxicity risk of upper GI bleeding, ulceration, obstruction, and perforation, but it does improve GI-OAR sparing in the low-intermediate dose range (below 30 GyE) while maintaining appropriate CTV and PTV coverage for localized pancreatic cancer without distant metastasis in comparison with IMRT and VMAT. The volumes of OARs irradiated varied among the three modalities. In two of the plans, because of a higher percentage of PTV overlap with GI-OARs, the PTV target coverage goal (*V*_90%_ ≥ 95%) was not met in order to completely abide by the OAR constraints with the best possible coverage. Despite that, the captivating conclusion could be derived from the plans that were created with full target coverage goals and could be extrapolated to new cases. This is the first NTCP model-based comparative study to quantitatively evaluate the risk of GI-OAR toxicity between proton and modulated photon radiation modalities in localized pancreatic cancer without distant metastasis.

Previous studies have accentuated the significance of lower and higher GI-OAR doses in their evaluation of radiation-related toxicity (5, 30–32). Severe bowel toxicity, such as perforation or obstruction and upper GI bleeding, depends on the volume in the high-dose (*V*_50GyE_) spectrum of DVHs, as suggested by the Quantitative Analyses of Normal Tissue Effect in Clinic (QUANTEC) and recent NTCP model prognosticating severe GI toxicity, derived from multiple-dose fractionation regimens (5, 33–35). In our study, the observed dosimetric differences in the *D*_max_ and *V*_50GyE_ for the stomach, duodenum, small bowel, and stoduo were statistically significant with the 3D-PSPBT plan in comparison with the IMRT and VMAT plans. However, in our study, 3D-PSPBT results in minimal NTCP reduction and has less potential to substantially reduce the toxicity risk of the upper GI bleeding, ulceration, obstruction, and perforation endpoints in comparison with IMRT and VMAT.

Acute GI toxicity endpoints such as radiation-induced nausea, vomiting, and diarrhea have been reported to occur in 20–70% of patients treated with upper abdominal irradiation (21, 36). No NTCP models have yet been defined so far for these endpoints, but some evidence suggests that volumes receiving low-to-intermediate dose range between 15 and 30 GyE may be predictive of acute nausea, vomiting, and diarrhea (5, 16, 19, 30, 37). The 3D-PSPBT plan resulted in a significantly reduced dose to GI-OARs in the low–intermediate dose range (below 30 GyE) than did the IMRT and VMAT plans, as shown in Table 3 and Figures 3C–E. The characteristic of the proton, together with its ability for several beam arrangements, produces a lower integral dose. A large GI-OAR volume receives a lower dose of radiation, but the most substantial dissimilarity appears above the 30-GyE dose area of the DVH between all three plans, and one clinical significance may be that 3D-PSPBT provides a method for improving the therapeutic ratio.

Our study has several limitations. A potential limitation of our research study is the use of photon-derived tissue NTCP models. Although clinical substantiation of these models was beyond the scope of this study, the relative NTCP comparisons made in this study should still be meaningful. Until randomized clinical comparisons of proton and modulated photon radiations are available, calculating NTCPs for toxicity assessments is an effective tool for comparing newly developed technique and treatment plan comparisons. The NTCP model selected in our study was generated based on similar patient cohorts and treatment for upper GI tumors. Our study did not consider the impact of proton variable RBE with interpatient variability of α/β and the composition of 3D-PSPBT fields (38, 39). Thus, cautious interpretation of the results of this study is essential because NTCP may have been affected by model uncertainties and the variable RBE of protons.

The conformity of the passive scattering technique is “2^1/2^D” in comparison with IMRT and VMAT planning since the PM and DM will have a similar shape, and its conformity is based on the CS. Thus, the passive scattering technique may hinder the full potential of proton beam therapy. The ability to spare normal tissues in high-dose areas apart from the Bragg peak region is limited because the lateral penumbra size with the passive scattering technique is similar to that of the photon, and it increases with target depth (16). A proton beam scanning (PBS) and intensity-modulated proton therapy (IMPT) could provide a much better comparison with the IMRT and VMAT plans. The studies by Ding et al. compared 3D-CRT *vs*. IMRT *vs*. 3D-PSPBT *vs*. PBS, and Jethwa et al. compared VMAT *vs*. robust multifield optimized (MFO) IMPT using 50.4 Gy of radiation dose in pancreatic cancer. These studies have reported that the PBS and robust MFO IMPT technique can lower the *D*_mean_ to the kidney and liver and can substantially reduce radiation exposure to GI-OARs in comparison with the 3D-CRT, IMRT, VMAT, and 3D-PSPBT techniques (40, 41).

All three plans were compared *in silico* by using an idealized treatment model in which the organ motion was not considered. Since the stomach and small bowel are expansible and movable, identifying the precise dose–volume constraints is quite challenging (42). Hence, image guidance with an adaptive treatment strategy is essential. However, the organ motion and respiration biases are common among patients who receive modulated photon or proton therapy and, thus, do not undermine the comparison of GI-OAR DVHs.

The proton dosimetry may be further improved by using the existing and future techniques that have not been considered in the present study. Lateral conformity can be enhanced by using PBS collimation, and a better dose deposition can be achieved by reducing the spot size in PBS (43). Future studies with calculation of the proton plans by taking the variable RBE of the proton into account will allow better comparisons between proton plans and with photon plans (44). The results of our study may provide the rationale for future research to investigate the benefits of 3D-PSPBT compared with modulated photon radiation in decreasing GI-OAR-related toxicity in patients with localized pancreatic cancer without distant metastasis treated with CRT.

## Conclusion

Our study showed that all three techniques provided adequate CTV and PTV coverages. 3D-PSPBT decreased the volume of GI-OARs receiving radiation doses at 50 GyE and the highest dose region. However, as per NTCP reduction, 3D-PSPBT does not have the potential to reduce radiation-related upper GI bleeding, ulceration, obstruction, or perforation in comparison with IMRT and VMAT. The 3D-PSPBT plan delivers a low-to-intermediate dose to lesser volumes of GI-OARs in comparison with the IMRT and VMAT plans and has the potential to reduce dose-limiting nausea, vomiting, and diarrhea. Future comparative clinical trials may determine the relative clinical significance of these phenomena.

## Data Availability Statement

All datasets generated for this study are included in the article/supplementary material.

## Ethics Statement

The studies involving human participants were reviewed and approved by National Cancer Center Hospital East (NCCHE) Institute Research Ethics Committee (Reference number: 2017-440). The patients/participants provided their written informed consent to participate in this study.

## Author Contributions

VR collected the patients' clinical data. TT and TR performed the treatment plans. VR and HH performed the data analysis. NN, SZ, AM, YH, KH, HB, TAr, HO, MN, MO, and YB suggested corrections and/or improvements. TAk performed major revision. All the authors have read and approved the manuscript and agreed to its submission.

## Conflict of Interest

The authors declare that the research was conducted in the absence of any commercial or financial relationships that could be construed as a potential conflict of interest.
